# Effects of Extracorporeal Shock Wave Combined with Vivaphototherapy on Blood Perfusion, Inflammatory Response, and Prognosis in Burn Patients

**DOI:** 10.1155/2022/1386875

**Published:** 2022-03-25

**Authors:** Jun Chen, Jianwei Nie

**Affiliations:** ^1^Wound Repair Department, The Second Affiliated Hospital of Fujian Traditional Chinese Medical University, Fuzhou, Fujian 350003, China; ^2^Department of Dermatology, Chiping District People's Hospital, Liaocheng, Shandong 252100, China

## Abstract

**Objective:**

To investigate the effect of extracorporeal shock wave treatment (ESWT) combined with water-filtered infrared-A (wIRA) therapy on pain, blood perfusion, and inflammatory response in burn patients.

**Methods:**

A total of 120 burn patients treated in our hospital from May 2019 to June 2021 were selected and randomly divided into observation group (*n* = 60) and control group (*n* = 60). The control group was treated with wIRA, and the observation group was treated with ESWT combined with wIRA. The hospitalization conditions of the two groups were observed; the visual analogue scale (VAS) was used to evaluate the pain on the 1st, 7th, and 14th days of treatment in the two groups; the blood perfusion was compared between the two groups; the levels of cerebral neuropeptide (NPY), 5-serotonin (5-HT), prostaglandin E2 (PGE2), C-reactive protein (CRP), interleukin-10 (IL-10), tumor necrosis factor-*α* (TNF-*α*), serum intercellular adhesion molecule-1 (sICAM-1), soluble-triggering receptor expressed myeloidcells-1 (sTREM-1), and soluble hemoglobin scavenger receptor (sCD163) were measured. Modified Vancouver Scar Scale (mVSS) was used to evaluate the wound scar at 3 and 6 months after the end of treatment.

**Results:**

The wound healing rate in the observation group was significantly higher than that in the control group, and the wound healing time and hospitalization time were significantly shorter than that in the control group (*P* < 0.05). On the 7th and 14th days of treatment, the VAS scores of the observation group were significantly lower than those of the control group (*P* < 0.05). On 1st, 7th, and 14th days of treatment, the blood perfusion volume in the observation group was significantly higher than that in the control group (*P* < 0.05). The scar scores in the observation group at 3 months and 6 months after treatment were significantly lower than those in the control group (*P* < 0.05). After treatment, the levels of NPY, 5-HT, PGE2, CRP, IL-10, TNF-*α*, sICAM-1, sTREM-1, and sCD163 in the observation group were improved more than those in the control group, and the differences were statistically significant (*P* < 0.05).

**Conclusion:**

ESWT combined with wIRA therapy can effectively improve the hospitalization situation of burn patients, relieve pain, improve blood perfusion, reduce scar hyperplasia, reduce inflammation, and have a good therapeutic effect.

## 1. Introduction

Burns are common clinical traumas, including flame burns, chemical burns, and electrical burns. Those with deep burns have severe tissue damage, which can even damage subcutaneous muscle tissue or bone. In addition, bacterial infection often occurs on burn wounds, which makes it difficult to heal and causes serious dysfunction, which can seriously affect patients' quality of life [1–3]. At present, free skin grafting is mostly used in clinical treatment of deep burn wounds. Regular high pressure dressing change after skin grafting can promote wound healing [4]. However, due to complications such as skin graft displacement, wound infection, and wound exudation, the overall effect of free skin grafting is not good. Extracorporeal shock wave treatment (ESWT) is an auxiliary measure for wound treatment, and its mechanism of action is not yet clear. ESWT can promote wound angiogenesis, stimulate wound cell proliferation and differentiation, increase tissue blood supply, and inhibit inflammation. As an adjuvant therapy for wound therapy, ESWT has the advantages of safety, noninvasive, effective, and easy to operate. The sound energy acting on the body can be converted into mechanical stimulation and promote wound healing by affecting the interaction between molecules and cells. Water-filtered infrared-A (wIRA) system filters the light energy in the wavelength band that is easy to produce thermal effect in the epidermis, retains the light energy in the wavelength band that patients can tolerate and has therapeutic value, and can increase the local tissue temperature of patients. At the same time, it will not overheat the patient's skin, which can effectively regulate the patient's tissue perfusion and oxygenation metabolism, improve the content of immunoglobulin and albumin in patients, and effectively improve the actual condition of patients. Previous studies have shown that IL-10, CRP, and TNF-*α* are involved in the inflammatory response of burn patients [5]. We speculate that ESWT combined with wIRA will have a positive impact on the prognosis of burn patients. Serum intercellular adhesion molecule-1 (sICAM-1) is a member of the immunoglobulin superfamily of cell adhesion molecules and is involved in regulating the development and differentiation of tissue cells, inflammation, immune response, wound repair, coagulation, etc. [6]. Soluble-triggering receptor expressed myeloid cells-1 (sTREM-1) is produced by myeloid cells and is involved in the immune response of the body [7]. Soluble hemoglobin scavenger receptor (sCD163) can promote the release of inflammation-related factors and promote inflammatory response [8]. Serum sICAM-1, sTREM-1, and sCD163 levels in burn patients are associated with infection complicated by sepsis. The purpose of this study was to investigate the effects of ESWT combined with wIRA therapy on pain, blood perfusion, and inflammatory response in burn patients. The results are reported as follows.

## 2. Materials and Methods

### 2.1. General Information

A total of 120 burn patients treated in our hospital from May 2019 to June 2021 were selected and randomly divided into observation group and control group, with 60 cases in each group. In the observation group, there were 36 males and 24 females, aged ranged from 24 to 45 years, with an average of 35.07 ± 3.82 years. The burned area was 15.04~21.05 cm^2^, with an average of 17.89 ± 1.27 cm^2^. There were 28 patients with flame burns, 19 with boiling fluid burns, and 13 with chemical burns. In the control group, there were 32 males and 28 females, aged ranged from 25 to 43 years, with an average of 35.38 ± 3.45 years. The burned area was 14.75-20.22 cm^2^, with an average of 17.50 ± 1.20 cm^2^. The causes of burn are as follows: flame burn in 28 cases, boiling liquid burn in 19 cases, and chemical burn in 13 cases. The general data of the two groups were comparable (*P* > 0.05). This study was approved by the hospital ethics committee. The ethical approval number is: reg. No. 2022003. All patients enrolled in this study were informed and signed the informed consent.

### 2.2. Inclusion Criteria

① All patients had second-degree burns on the body surface. There are two types of second-degree burns: superficial second-degree burns and deep second-degree burns. The superficial II degree means that the blisters on the surface of the burn are not easy to fall off, the surrounding area is slightly red and swollen, and the pain sensation is more sensitive. Deep II degree means that the wound surface has no blisters or the blisters are easy to fall off, the wound surface is red and white, and the pain sensation is sluggish. ② There was no compound injury. ③ All patients volunteered to participate in the study.

### 2.3. Exclusion Criteria

Exclusion criteria are as follows: ① patients with severe underlying diseases; ② patients with severe burns or inhalation injury; ③ patients with severe shock; ④ patients with coagulation dysfunction; ⑤ patients with immune diseases; ⑥ patients with serious organ dysfunction such as heart, liver, and kidney dysfunction; and ⑦ patients with consciousness disorders.

### 2.4. Methods

Both groups were given routine treatment such as anti-infection, fluid rehydration, nutritional support, correction of water, and electrolyte imbalance and acidosis. The control group was treated with wIRA, and the observation group was treated with ESWT combined with wIRA.

#### 2.4.1. wIRA Therapy

Routine dressing change was carried out, the outer dressing was removed, and the wound was rinsed and cleaned with physiological saline. The operator explained the precautions for light and heat protection and wore protective clothing and eye protection and used wIRA (Hydrosun TM 750, Beijing Haite Technology Co., LTD CHN) for radiation treatment. The light source of the therapeutic instrument was 25 cm away from the skin, the wavelength was adjusted to 0.56~1.40 μm, and the power was 750~780 W. Each irradiation was 20 min, once a day.

#### 2.4.2. ESWT

Extracorporeal shock wave therapy machine (MP-100, STORZ, SUI) was used for treatment. The treatment pressure was set to 1.8-2.6 bar, the frequency was set to 10 Hz, the handle pressure was moderate, the shock dose was 2000 times, and the interval between two treatments was 7 days.

### 2.5. Observation Indicators

① For comparison of hospitalization between the two groups, the wound healing rate, wound healing time, and hospital stay were compared between the two groups after 7 days of treatment. Wound healing rate = (original wound area − existing wound area)/original wound area × 100%. Wound healing time refers to the time of complete epithelialization of the wound. ② For pain score, visual analog scale (VAS) [9] was used to evaluate the pain degree of both groups before and after treatment. The total score was 0-10 points, 1-3 points were considered as mild pain, 4-6 points were considered as moderate pain, and 7-10 points were considered as severe pain. The higher the score was, the more severe the pain symptoms were. VAS scores were performed on the 1st, 7th, and 14th days of treatment, respectively. ③ For level of pain mediators, 5 ml of fasting venous blood was taken from the two groups, which was left standing and centrifuged at 3000 r/min for 15 min; then, the serum of the patients was separated and stored at -30°C for testing. The levels of neuropeptide (NPY), 5-hydroxytryptamine (5-HT), and prostaglandin E2 (PGE2) in brain were determined by enzyme-linked immunosorbent assay. ④ For blood perfusion, the blood perfusion in the same burn site before and after treatment was measured by the Laser Doppler Flow Imager (MOOR, LDI2, UK) in the two groups, and the instrument should be kept perpendicular to the burn site. ⑤ For comparison of scar score between the two groups, the patients in the two groups were followed up by telephone follow-up and monthly return visit for 6 months. The Modified Vancouver Scar Scale (mVSS) [10] was used to evaluate the scar situation of the two groups at 3 and 6 months after the end of treatment, and the scoring items included color (0 ~ 3 points), thickness (0 ~ 4 points), vascular distribution (0 ~ 3 points), and softness (0 ~ 5 points). The total score was 0 ~ 15 points, and the higher the score was, the more serious the scar was. ⑥ For levels of inflammatory factors, the serum to be measured was collected, the levels of C-reactive protein (CRP) were determined by immunoturbidimetry, and the levels of interleukin-10 (IL-10) and tumor necrosis factor-*α* (TNF-*α*) were determined by enzyme-linked immunosorbent assay. ⑦ For levels of sICAM-1, sTREM-1, and sCD163, the serum to be measured was taken, and the serum sICAM-1, sTREM-1, and sCD163 levels were determined by enzyme-linked immunosorbent assay.

### 2.6. Statistical Methods

The SPSS 20.0 statistical software was used to analyze the obtained data, measurement data were expressed as $\bar{x}\pm s$, independent sample *t*-test was used for comparison between groups, and paired *t*-test was used for comparison before and after treatment within groups. Count data were expressed as frequency and composition ratio, and *χ*^2^ test was performed, and *P* < 0.05 indicated that the difference was statistically significant.

## 3. Results

### 3.1. Comparison of Hospitalization Conditions between the Two Groups

The wound healing rate in the observation group was higher than that in the control group, and the wound healing time and hospitalization time were shorter than that in the control group, with statistical significance (*P* < 0.05), see Table 1.

### 3.2. Comparison of VAS Scores between the Two Groups

On the 1st day of treatment, there was no significant difference in the VAS score between the two groups (*P* > 0.05). On the 7th and 14th days of the treatment, the VAS score of the observation group was lower than that of the control group, and the difference was statistically significant (*P* < 0.05), see Table 2.

### 3.3. Comparison of Pain Mediator Levels between the Two Groups

Before treatment, there were no significant differences in NYP, 5-HT, and PGE2 levels between the two groups (*P* > 0.05). After 7 days of treatment, the levels of NYP, 5-HT, and PGE2 in both groups decreased, and the observation group was lower than the control group; the differences were statistically significant (*P* < 0.05), see Table 3.

### 3.4. Comparison of Blood Perfusion Volume between the Two Groups

On 1st, 7th, and 14th of treatment, the blood perfusion volume in the observation group was higher than that in the control group, and the difference was statistically significant (*P* < 0.05), see Table 4.

### 3.5. Comparison of Scar Scores between the Two Groups

The scar scores in the observation group at 3 months and 6 months after treatment were lower than those in the control group, and the differences were statistically significant (*P* < 0.05), see Table 5.

### 3.6. Comparison of the Levels of Inflammatory Factors between the Two Groups

Before treatment, there was no significant difference in the levels of serum IL-10, CRP, and TNF-*α* between the two groups (*P* > 0.05). After 7 days of treatment, the levels of serum IL-10, CRP, and TNF-*α* in the two groups were decreased, and those in the observation group were lower than those in the observation group; the difference was statistically significant (*P* < 0.05), see Table 6.

### 3.7. Comparison of Serum sICAM-1, sTREM-1, and sCD163 Levels between the Two Groups

Before treatment, there was no significant difference in serum sICAM-1, sTREM-1, and sCD163 levels between the two groups (*P* > 0.05). After 7 days of treatment, the levels of sICAM-1, sTREM-1, and sCD163 in the two groups decreased, and those in the observation group were lower than those in the observation group; the difference was statistically significant, see Table 7.

## 4. Discussion

According to the mode of action, extracorporeal shock wave can be roughly divided into two types, namely, radiation-type and focused type, and can be divided into high energy and low energy according to the difference of energy flow density. There is no unified conclusion yet. ESWT was used to promote wound healing as early as 1990, but its mechanism of action has been studied in recent years [11]. The mechanism of ESWT promoting wound healing is relatively complex, which can increase tissue blood supply, promote wound angiogenesis, stimulate wound cell proliferation and differentiation, and inhibit early inflammatory response, etc. The details can be summarized as follows. ① For promoting wound angiogenesis, local blood circulation improvement is conducive to wound healing, and extracorporeal shock wave can promote the expression of VEGF through the superoxide pathway, promote angiogenesis by regulating the expression of nitric oxide, and improve tissue blood vessels. In addition, extracorporeal shock wave can also increase the expression of PECAM-1 and various specific factors of angiogenic pathway to promote angiogenesis. ESWT can induce angiogenesis in the wound by upregulating a variety of proangiogenic genes, chemokines, and cytokines; improve oxygenation and blood supply to the wound; and promote tissue regeneration. ② For increasing tissue blood perfusion, according to relevant studies, ESWT can increase the blood supply of rat skin flap [12], which may be related to the promotion of angiogenesis and revascularization. ③ For promoting tissue regeneration, the regeneration capacity of wound tissue can determine the speed of wound healing, and a variety of factors can affect the speed of wound healing. ESWT can accelerate the rate of reepithelialization of burn wounds and wounds at donor sites [13]. ④ For inhibiting early inflammatory response, the early moderate inflammatory response in burn patients is conducive to wound remodeling and wound healing, but the further development of excessive inflammatory response can become MODS and SIRS, which further threaten patients' lives. Therefore, effective control of excessive inflammatory response is very important to promote wound healing. ⑤ For anti-infection, pathogenic microbial infection is one of the main causes of wound nonhealing for a long time. ESWT can kill Staphylococcus aureus colonized in clinical wounds and inhibit bacterial proliferation through a variety of mechanisms to promote wound reproduction. ⑥ For promoting the mobilization of mesenchymal stem cells and endothelial progenitor cells to the wound surface, the process of wound healing and regeneration includes complex molecular and cytological mechanisms. Acute ischemia can affect the overexpression of chemokines and growth factors, promote the migration of endothelial progenitor cells, and reduce cell apoptosis. In addition, ESWT can promote the growth of bone marrow mesenchymal stem cells and osteoblast differentiation, which is conducive to tissue regeneration and vascular formation. The light of the wIRA system is filtered through the system, and the light energy in the wavelength band that is easy to produce thermal effect on the epidermis is filtered out, while the light energy in the 780~1400 nm wavelength band that has therapeutic effect and is tolerated by the patient is retained. It can transform the energy carried into the biological energy that can be used by human tissues, increasing oxygen supply, blood supply, temperature, etc. The instrument has the advantages of convenient use and safety.

In this study, the observation group was treated with ESWT combined with wIRA, while the control group was treated with wIRA. The wound healing rate of the observation group was higher than that of the control group, and the wound healing time and hospitalization time were shorter than those of the control group. These results indicate that ESWT combined with wIRA therapy can effectively promote the wound healing of burn patients and shorten their hospital stay, which may be because ESWT combined with wIRA therapy can play a synergic therapeutic effect and accelerate the wound healing of patients compared with wIRA therapy alone. In this study, the VAS scores of the observation group were lower than those of the control group on the 7th and 14th days of treatment. And after 7 days of treatment, the levels of NYP, 5-HT, and PGE2 in the observation group were significantly lower than those in the control group. The above results indicate that ESWT combined with wIRA therapy can effectively relieve pain in burn patients. NYP, 5-HT, and PGE2 are all pain-related mediators, among which NYP can promote cell membrane depolarization, enhance capillary and vascular excitability, and cause pain. 5-HT can be involved in the regulation of collective mood, body temperature, and pain sensation. PGE2 is a prostaglandin with pain-inducing effect. It indicates that ESWT can reduce the level of pain mediators, and its specific mechanism may be that extracorporeal shock wave produces energy gradient differences between tissues of different densities during the treatment process, which can inhibit the release of pain substances and reduce the sensitivity of pain nerves [14]. Previous studies have shown that ESWT can inhibit pain [15–17], which is consistent with the results of this study. The comparison of blood perfusion and scar score between the two groups showed that the blood perfusion of the observation group was higher than that of the control group at 1st, 7th, and 14th days of treatment, and the scar score of the observation group was lower than that of the control group at 3 and 6 months after treatment. These results indicate that ESWT combined with wIRA therapy can effectively improve blood perfusion and reduce scar hyperplasia in burn patients, which may be related to the effect of extracorporeal shock wave on promoting VEGF expression through superoxide pathway, promoting angiogenesis, and increasing blood perfusion.

Studies have shown that IL-10, CRP, and TNF-*α* are involved in the inflammatory response of burn patients [5]. In this study, after treatment, the levels of serum IL-10, CRP, and TNF-*α* in the observation group were lower than those in the control group, indicating that ESWT can effectively inhibit the early inflammatory response in burn patients, and its specific mechanism needs to be further explored. In this study, the wound healing rate of the observation group was higher than that of the control group. The wound healing time and hospital stay in the observation group were shorter than those in the control group. ESWT combined with wIRA in the treatment of burns shortens the hospital stay and improves the wound healing rate. It confirmed our previous conjecture.

sICAM-1 is a ligand of lymphocyte function-associated antigen-1 (LFA-1), which can be expressed in activated T cells, epithelial cells, monocytes, and keratinocytes and can mediate the adhesion between lymphocytes and endothelial cells. It is closely related to the infiltration, trans-endothelial, and adhesion of inflammatory cells. According to related studies, the serum sICAM-1 level in burn patients is significantly higher than that in healthy people, and its level is positively correlated with the severity of burns [18]. sTREM-1 belongs to the immunoglobulin family, which is related to the activation of the body's inflammatory response. The level of inflammatory response in burn patients is increased, and the patients are very prone to sepsis. sTREM-1 protein is closely related to the occurrence of sepsis and immune suppression of the body. According to research, sTREM-1 can activate the nuclear factor- (NF-) *κ*B signaling pathway through the phosphorylation cascade, promote the release of inflammatory factors, further trigger immunosuppression, and promote the occurrence of sepsis [19]. sCD163 is a soluble substance distributed in blood and tissue fluid. Burn patients may have elevated levels of inflammatory responses and immune abnormalities, resulting in excessive activation of monocyte-macrophage cells, which eventually leads to upregulation of sCD163 levels. High expression of sCD163 is an independent risk factor for sepsis in burn patients [20]. In this study, after treatment, the improvement of serum sICAM-1, sTREM-1, and sCD163 levels in the observation group was greater than that in the control group, indicating that ESWT can effectively regulate the levels of serum sICAM-1, sTREM-1, and sCD163, which may be related to the inhibition of early inflammatory response and anti-infection effect of ESWT.

In conclusion, the application of ESWT combined with wIRA in the treatment of burn patients can effectively relieve pain, promote wound healing, enhance blood perfusion, reduce scar hyperplasia, and relieve inflammation, which has clinical application value.

## Figures and Tables

**Table 1:** Comparison of hospitalization conditions between the two groups ($\bar{x}\pm s$).

Group	Wound healing rate (%)	Wound healing time (d)	Hospital stay (d)
Observation group (*n* = 60)	83.38 ± 9.42	13.97 ± 2.12	17.90 ± 2.50
Control group (*n* = 60)	69.23 ± 5.64	18.57 ± 2.89	20.37 ± 3.06
*t* value	9.982	9.937	4.835
*P* value	<0.001	<0.001	<0.001

**Table 2:** Comparison of VAS scores between the two groups ($\bar{x}\pm s$, points).

Group	1st day of treatment	7th day of treatment	14th day of treatment
Observation group (*n* = 60)	7.48 ± 1.52	3.20 ± 0.95^∗^	1.15 ± 0.63^∗^^#^
Control group (*n* = 60)	7.67 ± 1.64	5.02 ± 1.33^∗^	1.70 ± 0.62^∗^^#^
*t* value	0.634	8.583	4.812
*P* value	0.528	<0.001	<0.001

^∗^ indicated *P* < 0.05 when compared with 1st day of treatment; ^#^ indicated *P* < 0.05 when compared with 7th day of treatment.

**Table 3:** Comparison of pain mediator levels between the two groups ($\bar{x}\pm s$).

Group	NYP (μg/l)		5-HT (ng/l)		PGE2 (pg/ml)	
	Before treatment	7th day of treatment	Before treatment	7th day of treatment	Before treatment	7th day of treatment
Observation group (*n* = 60)	232.16 ± 21.29	137.17 ± 13.64^a^	222.45 ± 22.73	92.53 ± 9.30^a^	228.28 ± 25.48	135.89 ± 11.32^a^
Control group (*n* = 60)	236.40 ± 21.35	179.71 ± 17.33^a^	226.80 ± 15.89	135.94 ± 13.31^a^	227.33 ± 21.87	165.32 ± 17.50^a^
*t* value	1.090	14.946	1.214	20.704	0.473	10.938
*P* value	0.278	<0.001	0.227	<0.001	0.637	<0.001

^a^ indicated *P* < 0.05 when compared with the same group before treatment.

**Table 4:** Comparison of blood perfusion volume between the two groups.

Group	1st day of treatment	7th day of treatment	14th day of treatment
Observation group (*n* = 60)	0.49 ± 0.06	0.74 ± 0.09^∗^	0.87 ± 0.10^∗^^#^
Control group (*n* = 60)	0.27 ± 0.05	0.48 ± 0.05^∗^	0.63 ± 0.08^∗^^#^
*t* value	20.588	20.215	14.846
*P* value	<0.001	<0.001	<0.001

^∗^ indicated *P* < 0.05 when compared with 1st day of treatment; ^#^ indicated *P* < 0.05 when compared with 7th day of treatment.

**Table 5:** Comparison of scar scores between the two groups ($\bar{x}\pm s$, points).

Group	3 months after treatment	6 months after treatment
Observation group (*n* = 60)	10.42 ± 1.67	5.42 ± 1.57^c^
Control group (*n* = 60)	12.68 ± 1.40	7.93 ± 1.89^c^
*t* value	8.066	7.824
*P* value	<0.001	<0.001

^c^ indicated *P* < 0.05 when compared with 3 months after treatment.

**Table 6:** Comparison of the levels of inflammatory factors between the two groups ($\bar{x}\pm s$).

Group	IL-10 (pg/ml)		CRP (mg/l)		TNF-*α* (μg/ml)	
	Before treatment	7th day of treatment	Before treatment	7th day of treatment	Before treatment	7th day of treatment
Observation group (*n* = 60)	29.01 ± 5.11	15.34 ± 3.80^a^	12.91 ± 3.23	30.38 ± 3.53^a^	183.72 ± 24.79	94.76 ± 53.27^a^
Control group (*n* = 60)	28.49 ± 4.55	18.49 ± 5.02^a^	12.61 ± 2.32	50.18 ± 9.92^a^	184.99 ± 25.69	132.66 ± 22.40^a^
*t* value	0.598	3.873	0.582	14.565	0.277	5.080
*P* value	0.551	<0.001	0.562	<0.001	0.783	<0.001

^a^ indicated *P* < 0.05 when compared with the same group before treatment.

**Table 7:** Comparison of serum sICAM-1, sTREM-1, and sCD163 levels between the two groups ($\bar{x}\pm s$).

Group	sICAM-1 (ng/ml)		sTREM-1 (pg/ml)		sCD163 (ng/ml)	
	Before treatment	7th day of treatment	Before treatment	7th day of treatment	Before treatment	7th day of treatment
Observation group (*n* = 60)	952.39 ± 126.02	680.23 ± 136.47^a^	85.78 ± 9.97	57.83 ± 6.91^a^	66.78 ± 8.19	41.26 ± 6.83^a^
Control group (*n* = 60)	927.50 ± 101.79	775.91 ± 101.38^a^	84.71 ± 8.07	72.15 ± 7.48^a^	67.62 ± 7.34	54.42 ± 5.35^a^
*t* value	1.190	4.359	0.641	10.890	0.592	11.736
*P* value	0.236	<0.001	0.523	<0.001	0.555	<0.001

^a^ indicated *P* < 0.05 when compared with the same group before treatment.

## Data Availability

The labeled datasets used to support the findings of this study are available from the corresponding author upon request.
